This article has been retracted.

# Real-Time Monitoring of Intraocular Pressure in Glaucoma Patients Using Wearable Mobile Medicine Devices

**DOI:** 10.1155/2022/2271937

**Published:** 2022-03-28

**Authors:** Xiangwen Yuan, Jiabin Zhang

**Affiliations:** Department of Ophthalmology, Jinan People's Hospital Shandong, Jinan 271100, China

## Abstract

Glaucoma is caused by excessive aqueous humor in the eye, resulting in a continuous or intermittent increase of intraocular pressure, which exceeds the tolerance of the eyeball and damages the optic nerve. Existing treatments for glaucoma do not work well or have significant side effects. Intraocular pressure signal is a very important physiological signal that needs real-time and accurate monitoring in glaucoma patients, especially in severe glaucoma patients. Therefore, long-term, real-time, and accurate monitoring of intraocular pressure is of great significance for the diagnosis and treatment of glaucoma patients. The use of wearable devices for real-time ocular diagnosis and treatment of glaucoma patients is an effective approach. However, the current commonly used intraocular pressure measurement and monitoring technology is difficult to meet the diagnosis and monitoring needs of glaucoma patients in terms of size, measurement accuracy, power consumption, and intelligence. Therefore, facing the needs of glaucoma disease treatment, this topic studies an implantable flexible intraocular pressure sensor for long-term continuous monitoring of intraocular pressure in glaucoma patients and mainly focuses on the working principle, structural design, process fabrication, measurement and control system, characterization, and performance test of the intraocular pressure sensor. It is of great significance for personalized and accurate treatment of glaucoma patients.

## 1. Introduction

Glaucoma is a serious and irreversible chronic ophthalmic disease that causes blindness. Its pathogenesis is mainly that the increase of pathological intraocular pressure (IOP) exceeds the bearing capacity of intraocular tissue, resulting in the damage of optic nerve and loss of visual function [1]. According to statistics, glaucoma is one of the eye diseases with the largest number of human blindness. There are more than 60 million glaucoma patients in the world. It was predicted that there would be 80 million glaucoma patients by 2020, and China is one of the countries with the largest number of glaucoma patients [2]. Although glaucoma cannot be completely cured, early prevention and timely treatment of glaucoma are of great significance to the patient's family and society.

The optic nerve damage of glaucoma is mainly attributed to intraocular pressure [3]. Intraocular pressure is the pressure exerted by the contents of the eyeball on the inner wall of the eyeball. The dynamic balance of intraocular aqueous circulation is one of the biggest factors affecting the fluctuation of intraocular pressure [4]. Some studies have shown that long-term intraocular pressure fluctuation is an important index of glaucomatous visual impairment, and greater intraocular pressure fluctuation will lead to greater visual field defects. The pathological intraocular pressure of glaucoma patients fluctuates for a long term [5]. By analyzing the fluctuation curve of intraocular pressure, it is found that the peak intraocular pressure of most patients is not in the time period of working in the hospital during the day. At present, the actual situation is that patients go to the hospital to detect intraocular pressure every few hours, which affects not only their rest but also the determination of accurate peak, valley, and fluctuation values, which is very unfavorable to the accurate diagnosis of glaucoma [6]. Similarly, real-time and accurate intraocular pressure data also play an important guiding role in the determination of personalized treatment schemes such as dose and time of administration for glaucoma patients. Therefore, real-time continuous and accurate monitoring of intraocular pressure is of great significance for the diagnosis and treatment of glaucoma patients, especially severe glaucoma patients [7].

The measurement of intraocular pressure is an important index for the diagnosis and treatment of ophthalmic diseases. At the same time, it is also particularly important for the diagnosis of glaucoma and the determination of personalized treatment plan. The measured value of intraocular pressure will be different due to different measurement principles and methods. At present, the measurement of intraocular pressure can be performed by using various intraocular pressure measuring instruments [8]. The commonly used intraocular pressure meters in clinics include flattening type, indentation type, and noncontact type. Although the measurement accuracy of GAT can reach 0.5 mmHg, the changes of central corneal thickness and corneal curvature will seriously affect the measurement results. Another disadvantage of GAT is that it can only measure intraocular pressure at a specific time during the day [9]. A typical indentation tonometer is used to indirectly measure the intraocular pressure value according to the degree of central corneal indentation caused by a certain external force. The advantages of an indentation tonometer are relatively simple structure and simple operation. However, it also has some disadvantages, such as cross infection and large measurement error. The measurement principle of noncontact tonometry (NCT) is to flatten the cornea to a certain area by air force. This method does not need direct contact with the cornea, does not need anesthetic, and reduces the probability of corneal infection. Therefore, it is suitable for screening glaucoma. However, an NCT tonometer also has some disadvantages, such as unable to accurately measure the intraocular pressure of patients with corneal lesions [10].

In recent years, with the continuous in-depth research on the principles and methods of intraocular pressure measurement, more and more new portable tonometers appear in front of people. However, some existing intraocular pressure measuring instruments improve the influence of cornea and other related factors on intraocular pressure measurement to a certain extent. However, due to the high cost of testing instruments and inapplicability of repeated measurements, it is still unable to achieve long-term continuous and accurate monitoring of intraocular pressure. In view of the above-mentioned problems [11], there is an urgent need to develop a sensor that can continuously monitor intraocular pressure in real time for the diagnosis and treatment of glaucoma patients, especially severe glaucoma patients. The complete intraocular pressure data obtained through long-term continuous intraocular pressure measurement can help doctors fully understand the patient's intraocular pressure fluctuation and make a more objective diagnosis [12]. The main contribution of this paper is to establish a measurement and control system that simulates the in vivo IOP environment. Its main function is to test the performance of sensors and simulate the experiments of in vitro IOP testing. The in vitro simulated IOP measurement and control system mainly consists of an environmental control module, a sealed chamber, and a signal processing module. The environmental control module mainly includes the control of pressure, temperature, and other environmental factors. The designed sealing chamber is a well-sealed container that can withstand certain pressure and is used to place the intraocular pressure sensor. The signal processing module includes the detection circuit and signal transmission module, which can amplify the signal sensed by the sensor. The effective combination of the three modules can meet the requirements of sensor performance testing and simulation of the in vivo intraocular pressure environment.

## 2. Related Work

### 2.1. Research Status of Implantable Intraocular Pressure Sensors

With the wide application of microelectromechanical systems (MEMSs) in implantable medical devices, more opportunities have been created for the treatment of human chronic diseases and the monitoring of physiological indexes [13]. For example, a cardiac pacemaker is the most frequently used implantable device in the world. For another example, brain electrodes developed in 1997 can effectively inhibit the tremor of Parkinson's disease by stimulating the depths of the brain. In addition, the development of electronics has gradually entered the post-molar era. Sensors and actuators focus not only on the development of MEMSs but also on the diversification of functions. Now, more and more implantable pressure sensors are widely used in the monitoring of human physiological indexes, such as blood pressure, intracranial pressure, and intraocular pressure.

So far, many researchers have done relevant research on continuous intraocular pressure monitoring.  Figure 1 shows the classification of continuous intraocular pressure monitoring technology [14]. Intraocular pressure monitoring technology can be divided into wireless communication mode and wired communication mode according to the different communication modes inside and outside the body. Wireless communication technology is the main development trend of implantable medical devices, in which inductive coupling technology is a typical wireless communication technology. At the same time, inductive coupling technology can be divided into passive type and active type according to whether it needs to provide power supply. Therefore, according to the above classification, implantable intraocular pressure sensors can be roughly divided into two categories: wireless passive intraocular pressure sensors and wireless active intraocular pressure sensors [15]. The research status of the two types of implantable intraocular pressure sensors is introduced in detail below.

Wireless passive pressure sensors, on the one hand, use passive devices and, on the other hand, do not rely on battery power supply and wired interconnection technology communication. At the same time, they have the advantages of simple structure, small volume, and low power consumption. Therefore, they are widely used in complex environments. For example, implantable intraocular pressure sensors are a typical application [16]. However, one of the main disadvantages of wireless passive pressure sensors is that they cannot transmit signals at a long distance, so they are not suitable for the field of long-distance signal transmission. The basic principle of signal transmission of wireless passive implantable intraocular pressure sensors is that when the intraocular signal changes, the coupling inductance outside the eye also changes, and the changed intraocular pressure signal is detected by an external impedance meter [17]. In the 1960s, some researchers proposed a wireless passive implantable intraocular pressure sensor based on LC resonance for continuous measurement of intraocular pressure [18]. Subsequently, some researchers improved the principle of wireless passive implantable intraocular pressure sensors. For example, an implantable wireless passive intraocular pressure sensor based on SU-8. The sensor is composed of plane spiral coils, metal parallel plate capacitors, and SU-8 pressure-sensitive film. The whole intraocular pressure sensor is completely encapsulated in SU-8 stack with good biocompatibility, and there is a cavity structure inside. The intraocular pressure signal is obtained by measuring the phase frequency shift of the external coil impedance. The transmission distance between the sensor implanted in vivo and the signal received in vitro can reach 6 mm, the relative sensitivity of the sensor in air can reach 7035 ppm/mmHg, and the relative sensitivity in normal saline can reach 3770 ppm/mmHg [19].

Wireless active implantable intraocular pressure sensors, compared with wireless passive implantable intraocular pressure sensors, have the advantages of infinite active intraocular pressure sensors such as the transmission signal distance is longer, the function is more powerful, and the communication quality is higher. At the same time, they bring the problem that the intraocular pressure monitoring microsystem is more complex. A typical active implantable intraocular pressure sensor is usually composed of CMOS control circuit, batteries, and pressure-sensitive unit [20].

### 2.2. Glaucoma Patients and Eye Pressure Analysis

Glaucoma is caused by an increase in intraocular pressure due to excess fluid in the eye that exceeds the tolerance of the eye, resulting in acute pain, visual loss, and even blindness. This project is based on microelectronic integration technology to develop an in vivo intelligent microtherapy system that integrates automatic monitoring and drainage of intraocular pressure, which can automatically adjust the intraocular pressure to a comfortable value without discomfort after implantation. The system is divided into two parts: extraocular and intraocular. Since the system implanted in the eye needs to drive the micropump and to meet the requirements of long-term operation, the extraocular part provides electrical power to the intraocular part through wireless power supply [10]. The doctor can set the target IOP for the system according to the degree of optic nerve and visual field damage, and the IOP is automatically monitored and actively regulated to within the normal range by the micropump. At the same time, the monitored data of the working status of the intraocular device are transmitted to the medical control terminal [11], so that the medical control terminal can grasp the performance of the intraocular device in time and adjust and set a new target IOP according to whether the patient's visual field has progressed or not and further guide the related research in depth and finally regulate the intraocular pressure to make it at a normal level.

### 2.3. Wearable Devices

IOP monitoring at home for glaucoma patients is very important for early diagnosis and effective treatment of glaucoma disease. In this paper, we propose and implement a wearable IOP continuous monitoring terminal for glaucoma patients' home application. The wearable module is designed to prevent secondary damage to the eye by misuse, which improves the operability and safety of the device. The most convenient way of continuous IOP monitoring is continuous IOP monitoring at home. The current technical bottleneck is that the existing portable IOP meters are relatively simple to operate but still require some preliminary professional guidance and training. In addition, they are offline single IOP measurement devices, lacking automatic remote data transmission function, and the standardization of patient data recording cannot be guaranteed. Intelligent IoT technology provides an effective technical way to solve this technical bottleneck problem. In this paper, we address the shortcomings of existing portable IOP meters in terms of ease of operation and remote data transmission and focus on a wearable intelligent nondestructive access terminal with a rebound IOP meter as the IOP measurement unit, aiming to develop a wearable IOT terminal with one-button operation that can be used correctly without professional training.

### 2.4. Research Status of Flexible Pressure Sensors

Intraocular pressure sensors are a kind of pressure sensors with small range and high precision. However, most of the above-mentioned pressure sensors based on traditional cavity structure still restrict the development of implantable intraocular pressure sensors to a certain extent [21]. In recent years, with the rapid development of sensing technology and nanomaterials, a new type of micro nano structure flexible pressure sensor has emerged, and many researchers have been attracted to use this new type of micro nano sensitive structure to study small-scale and high-precision flexible pressure sensors [22]. For example, Professor Bao Zhenan of Stanford University [23] designed the capacitive pressure sensor made of pyramid microstructure, which has high sensitivity. Its sensitivity is 30 times that of general pressure sensors without microstructure, and the sensor can detect the weight of a 20 mg green fly. For example, the nano friction power generation device developed by Professor Wang Zhong-Lin using micro nano structure can not only realize the function of the pressure sensor sensing pressure change but also achieve the effect of automatic energy supply [24].

In the 1990s, Japanese scientists discovered multiwall carbon nanotubes [25]. This discovery has caused a worldwide upsurge of nanotechnology research. At present, some studies have directly used nanomaterials and micro nano manufacturing technology to make high-sensitivity micro pressure sensors. For example, Zhang Yu's research group of Suzhou Institute of Nanotechnology, Chinese Academy of Sciences, studied a piezoresistive pressure sensor made of single-wall carbon nanotubes (SWCNTs) and silk surface microstructure, which can detect the changes of small forces such as pulse beat and sound vibration [26]. In 2016, the research group successively proposed a capacitive pressure sensor made of lotus leaf surface microstructure and polystyrene (PS) microspheres [27]. Although the research on implantable intraocular pressure sensor based on micro nano contact-sensitive structure is still blank, according to the above research paper on micro pressure sensors based on nanomaterials and microstructure, we believe that it is very promising to use the pressure sensors based on micro nano contact structure for pressure measurement of small organs such as the eyeball.

### 2.5. Problems in Existing Research

From the above research status of implantable intraocular pressure sensors and flexible pressure sensors at home and abroad, at present, the implantable intraocular pressure sensors and flexible pressure sensors based on micro nano contact-sensitivity mechanism have made a lot of research progress in all aspects, but there are still the following problems [28]:

1. At present, most implantable intraocular pressure sensors adopt cavity pressure-sensitive structure. According to the analysis of principle, when the material is determined, the relatively small pressure detection of intraocular pressure needs to be realized by increasing the radial size of the cavity. Therefore, it is difficult to reduce the size and further improve the integration of small organs such as implanted eyeballs.
2. At present, the packaging method of implantable intraocular pressure sensors can meet the requirements of stability and biocompatibility of the implanted human body in a short time, but it is difficult to meet the requirements of long-term implantation for more than several years.
3. Although the flexible pressure sensors based on micro nano contact structure have the advantages of high sensitivity and fast response, their application field still have some limitations, especially in biomedical and implantable applications.
4. At present, the research of multifunctional measurement and control system dedicated to analog intraocular pressure signal detection is not perfect, so the measurement and control system of intraocular pressure sensors needs to be further studied.

## 3. Scheme and Analysis

Aiming at the serious fluctuation of intraocular pressure in patients with severe glaucoma and the existing problems of intraocular pressure monitoring, an implantable flexible intraocular pressure sensor based on micro nano contact-sensitivity mechanism is proposed in this paper. Through literature research and analysis, this paper summarizes the research status of implantable intraocular pressure sensors at home and abroad and mainly focuses on the sensor principle, structural design, technology, measurement and control system, characterization, and performance test of sensing devices.

### 3.1. Research Program

According to the definition of a sensor, it is a device that converts the sensed physical quantity, chemical quantity, and other information into a device convenient for measurement and signal transmission according to a certain law. Generally speaking, the electrical signal is easier to process and transmit, and most of the sensor devices convert the nonelectric quantity into electrical signal. Therefore, the implantable flexible intraocular pressure sensor studied in this paper is also a pressure sensor device that converts the intraocular pressure signal into an easy-to-process electrical signal.

The intraocular pressure sensor studied in this paper is an important part of the intraocular pressure control system. The block diagram of the whole intraocular pressure control system is presented in Figure 2.

The controlled object is the eyes of glaucoma patients, the detection part is the implantable intraocular pressure sensor, and the controller and actuator are patients and treatment means, respectively. When the intraocular pressure of glaucoma patients is too high, the intraocular pressure signal detected by the implantable intraocular pressure sensor can be compared with the normal intraocular pressure value, the signal of intraocular pressure change is transmitted to doctors and glaucoma patients, and thus they are informed to drain or take other effective treatment measures in time, so as to control the intraocular pressure value of patients within the normal intraocular pressure range. The use of implantable intraocular pressure sensor to continuously detect the intraocular pressure signal of glaucoma patients in real time can help patients and doctors take effective treatment measures in time to control the deterioration of severe glaucoma patients. At present, an implantable aqueous humor drainage device is widely used in the treatment of glaucoma, especially for patients with severe glaucoma; the implantable drainage device is an effective way to reduce intraocular pressure. In this paper, the flexible intraocular pressure sensor combined with drainage device was implanted into the patient's eyes. The function of the intraocular pressure sensor is to detect intraocular pressure, and the function of the drainage device is to drain the aqueous humor. When the patient's intraocular pressure increases due to too much aqueous humor, the intraocular pressure sensor detects the intraocular pressure value and transmits it to the patient and doctor, and then the patient and doctor lead out the aqueous humor through the drainage device according to the measured intraocular pressure information to achieve the effect of reducing intraocular pressure.

To meet the needs of micro pressure signal detection and implantable special applications, a capacitive flexible intraocular pressure sensor based on micro nano contact-sensitive structure is studied in this paper. The flexible capacitive pressure sensor with micro nano contact-sensitive structure is more prone to deformation after being subjected to force, not only the electrode plate spacing will change, but also the dielectric constant will change, so the sensitivity of the sensor can be improved. Among them, the research of sensor body mainly includes the structural design, manufacturing process, packaging process, characterization, and performance test of flexible pressure sensors based on micro nano contact-sensing mechanism. Firstly, according to the working principle and structural design of intraocular pressure sensors, the appropriate sensor process is studied and formulated. At the same time, the intraocular pressure sensor is characterized and tested by high-resolution characterization instruments and appropriate measurement and control systems. Finally, according to the results of sensor characterization and performance test, the structural design and process parameters of the sensor are further optimized, so as to obtain a high-performance implantable flexible intraocular pressure sensor.  Figure 3 is the schematic diagram of intraocular pressure signal detection and transmission. The transmission of intraocular pressure signal is divided into two parts. The intraocular implantable intraocular pressure sensor detects the change of intraocular pressure, converts the pressure signal sensed by the sensor into an easy-to-process electrical signal through an external detection circuit and signal processing module.

### 3.2. Working Principle and Structure Design of the Sensor

This chapter focuses on the body of flexible pressure sensors based on contact-sensitivity mechanism. In the aspect of sensor technology, the material selection and process fabrication of flexible pressure sensors with contact structure are studied. At the same time, the packaging technology of sensor devices is studied according to the demand of long-term implantation into the human body. In this paper, a flexible capacitive pressure sensor with micro nano contact structure is fabricated by micromachining technology.

Capacitive pressure sensors appeared in 1970s, which convert pressure change signal into capacitive signal. The working principle of typical capacitive pressure sensors is shown in Figure 4. MEMS capacitive sensors have the advantages of high sensitivity, small drift, and low power consumption. At the same time, they also have the disadvantages of parasitic capacitance, large input impedance, complex detection circuit, and sensitivity to electromagnetic interference.

A capacitive sensor is a sensor that converts the measured physical quantity into a capacitive signal. A typical capacitive sensor is an ideal parallel plate capacitance structure, which is composed of two parallel metal plates separated by dielectrics (insulating material). When the influence of edge electric field is ignored, the calculation formula of capacitance is as follows:

(1) $$\begin{array}{c} C=\frac{\varepsilon_{0}\varepsilon_{r}A}{\text{d}}, \end{array}$$

where *C* is the capacitance value, *ε*_0_ is the vacuum dielectric constant, *ε*_*r*_ is the relative dielectric constant, *d* is the spacing between two parallel plate electrodes, and *A* is the relative area of the parallel plate. It can be seen from the above formula that as long as any one of the three parameters *ε*_*r*_, *A*, and *d* changes, *C* can change. According to the variation of the above three parameters, capacitive sensors are divided into variable medium type, variable area type, and variable pole distance type. Taking the variable pole distance capacitive sensor (*C*=*f*(d)) as an example, when the pole plate spacing is displaced, the pole plate spacing changes from *d* to *d*+*δ* and the capacitance value of the sensor will also change accordingly:

(2) $$\begin{array}{c} C=\frac{\varepsilon_{0}\varepsilon_{r}A}{\text{d}+\delta }. \end{array}$$

The relationship between capacitance and displacement is nonlinear. At the same time, the Taylor expansion is used:

(3) $$\begin{array}{c} F\left({\text{d}}_{0}+\delta \right)=F\left({\text{d}}_{0}\right)+\delta \frac{\partial F\left({\text{d}}_{0}\right)}{\partial \text{d}}+\frac{\delta^{2}}{2}\frac{\partial F\left({\text{d}}_{0}\right)}{\partial {\text{d}}^{2}}+\cdots . \end{array}$$

Approximating the relationship between capacitance and displacement:

(4) $$\begin{array}{c} C\approx \frac{\varepsilon_{0}\varepsilon_{r}A}{\text{d}}\left(1-\frac{\delta }{\text{d}}+\frac{\delta^{2}}{{\text{d}}^{2}}\right). \end{array}$$

When the initial value of the plate spacing is much greater than the change of displacement, the quadratic term of equation (4) can be omitted to obtain the relationship between the displacement sensitivity and capacitance of the sensor:

(5) $$\begin{array}{c} S_{\text{d}}=\frac{\partial C}{\partial \text{d}}\approx -\frac{\varepsilon_{0}\varepsilon_{r}A}{{\text{d}}^{2}}. \end{array}$$

According to the above formula (5), to improve the sensitivity of the capacitive sensor, on the one hand, the material with high dielectric constant *ε*_*r*_ can be selected as the intermediate medium and, on the other hand, the distance *d* between the two plates can be reduced or the action area of the plates can be increased. Theoretically, designing a capacitive sensor with large area and small spacing (thin) plates can not only increase the initial value of the capacitive sensor but also make the plates more susceptible to stress and deformation, so as to improve the sensitivity of the sensor. However, in fact, the performance parameters of the capacitive pressure sensor are not independent. The change of one parameter will inevitably affect the other parameters. Therefore, this capacitive pressure sensor with large area and thin spacing parallel plate structure also has many disadvantages. For example, the thinner plate is more prone to fracture under stress and will also affect the performance parameters such as linearity of the sensor. The pressure sensor designed as a parallel plate capacitance structure with large area and thin spacing is difficult to be applied in practice, and it is more difficult to be applied to intraocular pressure measurement. Therefore, based on the parallel plate capacitance structure, a flexible capacitive pressure sensor based on micro nano contact structure is proposed for intraocular pressure measurement, further improving the sensitivity of the pressure sensor. Therefore, the pressure sensitivity of the sensing device can be expressed as follows:

(6) $$\begin{array}{c} S_{P}=\frac{\partial C}{\partial P}=\frac{\partial C}{\partial \text{d}}\cdot \frac{\partial \text{d}}{\partial P}+\frac{\partial C}{\partial \varepsilon_{r}}\cdot \frac{\partial \varepsilon_{r}}{\partial P}. \end{array}$$

According to formula (6), compared with the commonly used parallel plate or capacitive pressure sensor with cavity structure, when the flexible capacitive pressure sensor with micro nano contact-sensitive structure is subjected to pressure, in addition to the capacitance change caused by the distance between capacitive plates, the change of dielectric constant of the micro nano contact structure will further significantly cause the change of capacitance. The capacitive pressure sensor with micro nano contact-sensitive structure designed in this paper is mainly composed of a packaging layer, an electrode layer, a dielectric layer, a micro nano structure, and a substrate. Its structural principle diagram is shown in Figure 5.

### 3.3. Research on the Measurement and Control System of Intraocular Pressure Sensors

This chapter focuses on the measurement and control system of the sensor. Its main function is to test the performance of the pressure sensor and simulate the intraocular pressure measurement environment in vitro. The measurement and control system is mainly composed of a pressure loading part and capacitance signal detection part. The pressure loading part includes liquid, gaseous, and solid pressure loading forms, and the capacitance signal detection mainly includes the capacitance detection circuit and electronic measurement instrument. The sensor measurement and control system for analog intraocular pressure measurement is mainly composed of the environmental control module, sealed cavity, and signal processing module. The environment control module includes the control of pressure and temperature.

The signal of the capacitive sensor is generally small, but the change signal of micro capacitance is smaller, which adds great difficulty to the subsequent circuit processing. Therefore, it is of great significance to design an appropriate capacitance detection circuit for the detection of micro capacitance. There are four types of detection circuits of capacitive pressure sensors, namely oscillator detection circuit, resonant detection circuit, charge-discharge detection circuit, and AC bridge detection circuit. Based on the characteristics of the four conventional capacitance detection circuits introduced above, we summarize the advantages and disadvantages of the four conventional capacitance detection circuits in Table 1 with reference to relevant literature and experimental results [8, 9].

Compared with the traditional capacitance detection circuit, the integrated chip capacitance detection circuit has higher capacitance resolution, has stronger anti-interference ability, and is easy to convert into digital signals. Therefore, the integrated chip capacitance detection circuit is first selected to detect small capacitance. Through literature research and analysis, this paper focuses on two kinds of integrated chip capacitance detection circuits, namely, the capacitance detection circuit based on MS3110 chip and PCAP01 chip. Through the above analysis of MS3110 chip and PCAP01 chip, we reviewed the experimental results of related literature [10–12] and summarized the performance parameters of these two integrated chip capacitance detection methods, as shown in Table 2.

According to the performance comparison between MS3110 chip and PCAP01 chip in Table 2, both chips convert capacitance signal into voltage signal, and the capacitance detection resolution can reach the aF level, which can be used for the detection of small capacitance. The values of the capacitance sensor and reference capacitance should be in one order of magnitude as far as possible, which can reduce the gain offset and improve the measurement accuracy. The main work of this chapter is to establish the measurement and control system of the sensor. Firstly, the pressure loading part of the measurement and control system is designed and manufactured. Finally, the performance of the pressure sensor is stably tested through the debugged measurement and control system.

## 4. Experiments and Results

Human eye pressure fluctuates at different times of the day, and achieving continuous IOP monitoring plays an important role in the accurate diagnosis of glaucoma disease. Likewise, for the treatment of glaucoma patients, real-time monitoring of IOP throughout the day is even more important. Based on this, we conducted many experiments mainly on micro nano contact capacitive pressure sensors for further exploring the use of micro nano contact capacitive pressure sensors for real-time IOP monitoring in glaucoma patients.

In this chapter, the high-resolution characterization and testing of micro nano contact-sensitive structures involve the characterization of micro nano scale and flexible nonconductive structures. Therefore, high-resolution characterization instruments are needed to directly characterize the surface morphology and other parameters of micro nano contact-sensitive structures. The characterization results play an important role in analyzing the principle of micro nano contact-sensitive mechanism and improving the sensor process. The experimental environment of this paper is as follows—reagents: graphene oxide powder (99%, Aladdin), ascorbic acid (99%, Aladdin), multiwall carbon nanotubes (95%, Aladdin), deionized water, acrylamide (99%, Aladdin), SDS (99.0%, Aladdin), UPYHCEA, NaCl (99.0%, Aladdin), TEMED (99%, Aladdin), APS (98%, Aladdin); and instruments: LCR digital bridge, scanning electron microscope (SEM).

### 4.1. Performance Test of the Sensor

The established sensor measurement and control system is used to test the performance of the capacitive pressure sensor with pyramid microstructure, and the relationship curve between the capacitance and pressure of the sensor is obtained, as shown in Figure 6.

From the curve fitting results, it is concluded that the capacitance of the sensor is positively correlated with the pressure, and the capacitance increases rapidly with the pressure in a small range. When it exceeds a certain range, the capacitance increases slowly. The sensitivity of pressure sensor is a very important parameter in the performance index of pressure sensor.

(7) $$\begin{array}{c} S=\frac{\left(\Delta C/C_{0}\right)}{\Delta P}, \end{array}$$

where *P* is the applied pressure, Δ*P* is the change of pressure, *C*_0_ is the initial capacitance of the capacitive pressure sensor, Δ*C* is the change of capacitance, Δ*C*/*C*_0_ is the relative variation of capacitance, and *S* represents the sensitivity of the capacitive pressure sensor.  Figure 7 shows the relationship curve between the relative change of capacitance and pressure. According to the experimental data and formula (equation (7)), it is concluded that the sensitivity of the sensor with pyramid micro nano structure reaches 0.21/kPa.

This paper focuses on the performance of the micro nano contact capacitive pressure sensor made of carbon nanotubes, including the stability, repeatability, hysteresis, and sensitivity of the sensor. In order to ensure the reliability of the test data, the capacitive pressure sensor is tested by applying pressure and unloading pressure for many times under the same experimental conditions. In this paper, the impedance measuring instrument and PCAP01 capacitance detection circuit are used to detect the capacitance. The initial capacitance of the pressure sensor is 8.87 pF.  Figure 8 shows the relationship curve between the capacitance value and the pressure change after the capacitive pressure sensor is averaged for many times.

According to the definition of repeatability of the sensor, the inconsistency of the characteristic curve is obtained by continuously applying pressure or reducing pressure in the same direction. According to the analysis of the above experimental data, it is concluded that the capacitive pressure sensor has good repeatability, hysteresis, and stability. When a certain range is exceeded, the sensitivity of the sensor will gradually decrease with the increase of pressure. From the above experimental results, it is concluded that the micro nano contact capacitive pressure sensor made of multiwall carbon nanotubes has high sensitivity and is suitable for the measurement of micro pressure.

### 4.2. Result Analysis

The surface morphology characterization and performance test results of the multiwall carbon nanotube pressure sensor are analyzed. The sensitivity of the pressure sensor increases with the increase of pressure within a certain range. When it exceeds a certain range, the sensitivity of the sensor will decrease with the increase of pressure. In the small pressure range of the pressure sensor, the micro nano contact structure deforms greatly, resulting in a large change in the distance between the sensor plates and a large dielectric constant, so the sensitivity of the pressure sensor increases. When the pressure exceeds a certain range, the micro nano contact structure of the pressure sensor is not easy to deform, so the sensitivity of the pressure sensor will be reduced. At the same time, the sensitivity of pressure sensors with electrode layers made of other materials in relevant literature is analyzed and compared, as shown in Table 3.

From the characterization results of the surface morphology of the micro nano contact-sensitive structure of the above sensor, it can be seen that the surface morphology of pyramid microstructure is more regular than that of carbon nanotubes. According to the characterization and performance test results, although the performance of the pyramid microstructure capacitive pressure sensor fabricated by the single chip packaging process is not particularly ideal, this regular pyramid structure is controllable, which plays a very important role in further studying the sensitivity mechanism of the sensor with micro nano contact structure. Due to limited time, the performance of pyramid microstructure pressure sensors will be improved in the follow-up research.

In this chapter, the micro nano contact capacitive pressure sensor is characterized and tested. The surface morphology of micro nano contact structure was characterized by high-precision characterization and testing instruments. At the same time, the performance of the capacitive pressure sensor with micro nano contact structure is tested by using the established sensor measurement and control system, and the pressure response characteristics and temperature response characteristics of the capacitive pressure sensor are also tested.

## 5. Conclusion

An implantable intraocular pressure sensor that can monitor intraocular pressure accurately for a long term and in real time is of great significance for the diagnosis and treatment of glaucoma patients, especially severe glaucoma patients. Therefore, this paper focuses on the body and measurement and control system of implantable flexible intraocular pressure sensors. For the body of the sensor, this paper studies a capacitive pressure sensor based on micro nano contact-sensitivity mechanism for intraocular pressure measurement, mainly including the structural design and process research of the sensor. At the same time, in order to meet the requirements of the performance test of implantable flexible intraocular pressure sensor and in vitro simulation of intraocular pressure environment, the measurement and control system of the sensor is established in this paper. Using high-precision characterization and measurement instruments and the established measurement and control system to characterize and test the performance of capacitive pressure sensor based on micro nano contact structure is also the focus of this paper. Finally, according to the characterization and performance test results of the sensor, the sensor structure design, process flow, and measurement and control system are optimized. The experimental results show that the micro nano contact capacitive pressure sensor made of carbon nanotubes has good repeatability, hysteresis, and stability, with a sensitivity of 1.3/kPa and a response time of milliseconds to the load, and it is not easily affected by temperature.

The implantable flexible intraocular pressure sensor studied in this paper has been working towards implantable applications, including material selection, sensor principle, process fabrication, and in vitro simulated intraocular pressure measurement. The implantable flexible intraocular pressure sensor based on micro nano contact-sensitivity mechanism proposed in this paper will promote the application of this flexible microsensor in medical diagnosis and health monitoring. Due to limited time and knowledge, there are still some problems in the research process to be identified. These problems will be improved in follow-up research. In the future, we plan to conduct research on overly skin electronic and nanoscale pressure sensors for glaucoma treatment and detection.

## Figures and Tables

**Figure 1:** Classification of continuous intraocular pressure monitoring.

**Figure 2:** Block diagram of intraocular pressure control system.

**Figure 3:** Schematic diagram of intraocular pressure signal detection and transmission.

**Figure 4:** Schematic diagram of the working principle of a capacitive pressure sensor.

**Figure 5:** Structural principle diagram of the micro nano contact capacitive pressure sensor.

**Figure 6:** Input-output curve of the sensor.

**Figure 7:** Relation curve between relative variation of capacitance and pressure.

**Figure 8:** Input and output curve of the sensor after averaging.

**Table 1:** Advantages and disadvantages of the four traditional capacitance detection circuits.

Circuit type	Advantage	Shortcoming
ODC	Simple circuit principle	Poor stability
RDC	Wide frequency range	No real-time measurement
CDDC	High precision	No automatic balancing
ACBDC	Mild drift flow	Poor stability

**Table 2:** Performance comparison between MS3110 chip and PCAP01 chip.

Performance index	MS3110	PCAP01
CDR	4.0 aF	4.0 aF
CMR	250 fF	50 fF
OFR	500 ~ 8000 Hz	500 kHz
NSDV	True	True
WC	2.9 mA	4.0 *μA*

**Table 3:** Sensitivity comparison of pressure sensors made of different electrode materials.

Material	Electrode material	Sensitivity
PDMS	Au	4.0*∗*10^−4^
PDMS	Ag	3.6*∗*10^−3^
PDMS	Cu	1.8*∗*10^−3^
PDMS	ITO	2.0*∗*10^−2^
PDMS	Al	4.0*∗*10^−2^
PDMS	AgNW	0.124
PDMS	NWTU	1.3

## Data Availability

The data sets used during the current study are available from the corresponding author on reasonable request.
